# Efficacy and Safety of PD-1/PD-L1 Inhibitor Chemotherapy Combined with Lung Cancer Fang No. 1 in Relapsed and Refractory SCLC: A Retrospective Observational Study

**DOI:** 10.1155/2022/2848220

**Published:** 2022-05-09

**Authors:** Lihua Wang, Xiaoxia Lei, Xin Wang

**Affiliations:** ^1^Department of Respiratory Endology, People's Hospital of Dongxihu District, Wuhan, Hubei 430040, China; ^2^Second Ward, Department of Respiratory and Critical Care Medicine, Wuhan No. 1 Hospital, China; ^3^Department of Infectious Disease, Wuhan Asia General Hospital, China

## Abstract

**Background:**

Relapsed and refractory small cell lung cancer (SCLC) accounts for about 15% of all lung cancers. The prognosis of patients is poor. The 5-year survival rate is almost 0. The average survival time of patients who refuse to receive treatment is only 2-4 months. For patients with extensive-stage SCLC, the current first-line treatment regimens are mainly platinum-containing double-drug chemotherapy. Poside combined with cisplatin/carboplatin and irinotecan combined with cisplatin/carboplatin are commonly used clinical regimens for the treatment of patients with extensive-stage SCLC. Although SCLC is very sensitive to radiotherapy and chemotherapy, most patients will develop recurrence and metastasis after initial treatment. Therefore, it is necessary to study clinically effective therapeutic drugs for relapsed and refractory SCLC.

**Objective:**

To investigate the relationship between programmed death receptor-1 (programmed death receptor-1 (PD-1)) and programmed death receptor-ligand 1 (programmed death-ligand 1 (PD-L1)) inhibitors and Lung Cancer No. 1 efficacy and safety of Lung Cancer Fang No. 1 in the treatment of relapsed and refractory SCLC.

**Methods:**

80 patients with refractory SCLC were selected and randomly divided into control group and treatment group with 40 cases in each group. Among them, the control group received PD-1/PD-L1 inhibitor chemotherapy, and the treatment group received PD-1/PD-L1 inhibitor chemotherapy combined with Lung Cancer Fang No. 1 treatment. The differences in immune and tumor marker levels, clinical efficacy, and prognostic complications between the two groups before and after treatment were observed and compared.

**Results:**

Before treatment, there was no significant difference in clinical improvement between the two groups. After treatment, the clinical symptom scores and body weight changes in the treatment group were significantly improved. The clinical symptom scores in the treatment group were lower than those in the control group, but the body weight changes were higher than those in the control group. The difference was statistically significant (*P* < 0.05). Before treatment, there was no significant difference in the levels of tumor markers between the two groups. After treatment, the levels of CYFRA21-1, CA125, and VGEF in the treatment group were significantly lower than those in the control group, and the difference was statistically significant (*P* < 0.05). There was no significant difference in the immune level between the two groups before treatment (*P* > 0.05), while the differences in CD4+, CD3+, and CD4+/CD8+ after treatment were significant, and the treatment group was higher than the control group, with statistical significance (*P* < 0.05). After treatment, the clinical efficacy of the two groups was significantly improved. The DCR90.00% of the treatment group was significantly higher than that of the control group, 67.50%, and the difference was statistically significant (*P* < 0.05). The analysis of complications after treatment showed that fatigue, anorexia, hypertension, hand-foot syndrome, diarrhea, leukopenia, thrombocytopenia, and urinary protein in the treatment group were significantly lower than those in the control group, and the difference was statistically significant (*P* < 0.05).

**Conclusion:**

PD-1/PD-L1 inhibitor chemotherapy combined with Lung Cancer Fang No. 1 has a good and safe effect on SCLC patients. It has a good curative effect in improving the clinical symptoms of patients. It can stabilize the tumor, inhibit the development of lung cancer, improve the body's cellular immune function, adjust the level and expression of tumor markers, improve the body's material metabolism, and restore the balance of yin and yang in the body.

## 1. Introduction

The 2019 American Cancer Report pointed out that the incidence of lung cancer ranks second among malignant tumors, and the mortality rate ranks first [1]. SCLC is a very destructive and aggressive neuroendocrine tumor, accounting for approximately 15% to 20% of all lung cancers [2]. Compared with non-SCLC, SCLC has biological characteristics such as low degree of differentiation, high degree of malignancy, easy recurrence and metastasis, and poor prognosis. About 70% of SCLC patients are diagnosed at an advanced stage, and the overall 5-year survival rate is less than 10% [3]. For inoperable patients, the objective response rate of first-line platinum-containing doublet chemotherapy is higher, but more than 80% of patients will relapse within 2 years, and the median survival (OS) after relapse is only 4-5 months [4]. In recent years, immune checkpoint inhibitors have made important progress in the field of tumor treatment. PD − 1 (programmed death receptor − 1), an important immunosuppressive molecule, belongs to the immunoglobulin superfamily and is a membrane protein with 288 amino acid residues.Immunoregulation targeting PD − 1 has great significance in inhibiting tumors, infections, and autoimmune diseases and protecting organ transplantation survival.The ligand PD − L1 also acts as a target, as do corresponding antibodies.The expression of PD − L1 on tumor cells inhibits antitumor activity through the binding of PD − 1 to effect T cells. Immune checkpoint inhibitors represented by PD-1/PD-L1 inhibitors mainly act on various inhibitory signals such as PD-1/PD-L1. PD-1/PD-L1 inhibitors have achieved remarkable curative effect in various malignant tumors such as non-SCLC, liver cancer, bladder cancer, and head and neck squamous cell carcinoma, which brought a survival benefit to patients [5]. There are many adverse reactions of PD-1/PD-L1 inhibitor treatment, but the clinical application of Lung Cancer No. 1 has a significant effect, which can significantly improve clinical symptoms. The no. 1 prescription for lung cancer mainly consists of Codonopsis pilosula, Radix angelicae dahurica, and Atractylodes macrocephala, tonifying the spleen, invigorating qi, and reducing phlegm dampness, accompanied by anticancer. Fatigue syndrome has a significant curative effect, such as improving the quality of life, prolonging the life of patients, and improving immune function [6]. Based on this, we explored the efficacy and safety of PD-1/PD-L1 inhibitor chemotherapy combined with Lung Cancer Fang No. 1 in relapsed and refractory SCLC. The current research results are reported as follows.

## 2. Material and Methods

### 2.1. Research Object

In this study, patients and their families have been informed and signed informed consent. A total of 80 SCLC patients who were treated in our hospital from April 2018 to July 2021 were selected as the research subjects and divided into the control group and the treatment group with 40 cases in each group according to the random remainder method. Differences in general clinical data such as gender, age, and body mass index between the two groups had no effect on this study. For details, see Table 1.

### 2.2. Exclusion Criteria

Inclusion criteria: (i) all patients in this study met the diagnostic criteria for SCLC in the “Chinese Medical Association Lung Cancer Clinical Guidelines (2018 Edition)” [7] and (ii) the pathological diagnosis of SCLC and the Eastern Cooperative Oncology Group (ECOG) score [8]: 0-2 points, most of the patients have lost the opportunity of surgery and chemoradiotherapy or have definitely refused surgery and chemoradiotherapy, and the last chemotherapy time is more than 4 weeks; chest tightness, cough and asthma, expectoration, shortness of breath, sore back, weak knees, dizziness, tinnitus, aversion to cold, and micro and thin pulse; Karnofsky score (KP) quality of life above 50 points, no drug, and for food allergy, the patient is willing to accept the treatment of this program, can adhere to the medicine as prescribed by the doctor, and has good compliance.

Exclusion criteria: (i) patients with serious primary diseases such as heart, liver, kidney, hematopoietic system, and mental illness; pregnant and lactating women; and poor compliance; (ii) patients who are pregnant, may be pregnant, have no effective contraception, and are breastfeeding, due to other reasons; the researchers think that patients are not suitable for inclusion; and (iii) patients with underlying diseases such as severe diabetes, high blood pressure, heart disease, or serious infections who require hospitalization.

### 2.3. Nursing Intervention Methods

The control group received PD-1/PD-L1 inhibitor chemotherapy, namely, PD-1/PD-L1 inhibitor treatment, including 25 cases of nivolumab, 13 cases of pembrolizumab, 1 case of sintilimab, and 1 case of atezolizumab. Specific usage: pembrolizumab 2 mg/kg, once every 3 weeks; nivolumab 3 mg/kg, once every 2 weeks; sintilimab 200 mg, once every 3 weeks; and atezolizumab 1200 mg, once every 2 weeks. The treatment group was treated with Lung Cancer Fang No. 1 on the basis of the control group, namely, Codonopsis 9 g, Scutellaria 9 g, Atractylodes 9 g, Poria 15 g, Polyporus 15 g, Sunshine Maoren 5 g, Chenpi 9 g, Hedyotis diffusa 30 g, Houttuynia cordata Grass 30 g, and iron leaves 30 g. Decoction in water, 1 dose a day, 3 times a day. Add or subtract according to the disease, decoction into decoction, one dose per day, take 3 times. One month is one course of treatment, and the observation period is three courses of treatment.

### 2.4. Flow Cytometry

Flow cytometry (FCM) is a quantitative analysis of single cells at the functional level. The cells to be tested were stained into a single cell suspension and stained with antibodies labeled with specific fluorescent dyes. Under the irradiation of laser beam, the cells would produce scattered light and excitation fluorescence.

### 2.5. Observation Indicators

Symptoms include cough, expectoration of sputum, hemoptysis, chest tightness, fatigue, chest pain, and fever, which are divided into 4 grades according to clinical observation: asymptomatic 0 point, mild 1 point, moderate 2 points, and severe 3 points. The symptoms were recorded before and after treatment. CD4+, CD3+, and CD4+/CD8+ were detected by Beckman CytoFLEX flow cytometer. Efficacy evaluation criteria: the short-term efficacy was evaluated according to RECIST. The following are the efficacy evaluation criteria for solid tumors: complete remission (CR): all target lesions completely disappeared except for nodular disease. All target nodules must be reduced to normal size (short axis < 10 mm). All target lesions must be evaluated. Partial response (PR): the sum of the diameters of all measurable target lesions is ≥30% below baseline. The short diameter was used for the sum of target nodules, while the longest diameter was used for the sum of all other target lesions. All target lesions must be evaluated. Stable (SD): not eligible for CR, PR, or progression. All target lesions must be evaluated. Progression (PD): a 20% increase in the sum of the diameters of the measurable target lesions beyond the minimum sum observed (above baseline, if no reduction in the sum was observed during treatment), with a minimum absolute increase of 5 mm. Disease control rate (DCR) = (CR + PR + SD)cases/total cases × 100%.

### 2.6. Statistical Analysis

Use EpiData to enter all the data, and then use SPSS 25.0 to statistically process the data. The data needs to be entered into a computer database by a second person to ensure the completeness and accuracy of the data. *χ*^2^ test is used to express the count data as a percentage (%). For each parameter, data is mentioned as mean ± SD and statistically analysed by employing one-way ANOVA followed by Tukey's multiple comparison post hoc test. *P* < 0.05 is considered as statistically significant.

## 3. Results

### 3.1. General Data Comparison

The gender, average age, tumor diameter, pathological type, and other general data of the two groups of patients were compared by *t* test and chi-square test, and there was no significant difference (*P* > 0.05). See Table 1.

### 3.2. Clinical Improvement

Before treatment, there was no significant difference in the clinical improvement of the two groups of patients. After treatment, the clinical symptom scores and body weight changes of the treatment group were significantly improved. This difference was significant for academic comparison (*P* < 0.05). See Figure 1.

### 3.3. Comparison of Tumor Marker Levels

Before treatment, there was no significant difference in the levels of tumor markers between the two groups. After treatment, the levels of CYFRA21-1, CA125, and VGEF in the treatment group were significantly lower than those in the control group, and the difference was statistically significant (*P* < 0.05). See Figure 2.

### 3.4. Immune Level Comparison

The immune levels of the two groups of patients before treatment were comparable, and the CD4^+^, CD3^+^, and CD4^+^/CD8^+^ after treatment were significantly different, and the treatment group was higher than the control group, with statistical significance (*P* < 0.05). See Figure 3.

### 3.5. Comparison of Clinical Efficacy

After treatment, the clinical efficacy of the two groups was significantly improved. The DCR90.00% of the treatment group was significantly higher than that of the control group, 67.50%, and the difference was statistically significant (*P* < 0.05). See Figure 4.

### 3.6. Prognostic Complications

The analysis of complications after treatment showed that fatigue, anorexia, hypertension, hand-foot syndrome, diarrhea, leukopenia, thrombocytopenia, and urinary protein in the treatment group were significantly lower than those in the control group, and the difference was statistically significant (*P* < 0.05). See Figure 5.

## 4. Discussion

Modern medical treatment of relapsed and refractory SCLC mostly adopts comprehensive treatment methods such as surgery, chemotherapy, radiotherapy, and immunization. Drug resistance limits the clinical application of these methods [9]. Despite the continuous update of chemotherapy drugs and the continuous optimization of various combination treatment options of radiotherapy, chemotherapy, and surgery, the curative effect is still unsatisfactory. Therefore, how to make the curative effect of these treatment methods better and longer and how to reduce the damage to the human body caused by these treatment methods, so that patients can adhere to the treatment and improve the quality of life, is a difficult problem for Western medicine [10]. Traditional Chinese medicine treatment has great advantages and research value in these aspects. With the deepening of TCM's understanding of lung cancer and the continuous improvement of clinical efficacy, TCM and integrated TCM and Western medicine have a unique role and status in the comprehensive treatment of lung cancer [11–13]. In this study, the use of Lung Cancer No. 1 formula in the treatment of SCLC can significantly improve the symptoms of patients, improve the immune function of the body, and has a certain synergistic effect. Fang Lung Cancer No. 1 can invigorate the kidney and nourish the marrow, nourish both yin and yang, and have the effect of nourishing qi, nourishing essence, and strengthening the body. Constrain it, so it is used to support the right without helping the evil, and eliminating the accumulation without hurting the right [14]. At the same time, the efficacy of traditional Chinese medicine and modern pharmacological research also provided the basis for the formulation mechanism of Lung Cancer No. 1 formula. Lung Cancer No. 1 recipe is composed of American ginseng, white mustard seed, Houttuynia cordata, chicken Neijin, and other traditional Chinese medicines. In the recipe, American ginseng is used to nourish qi and nourish yin, clear fire, and promote fluid, so as to improve the patient's low physical strength and fatigue after illness [15–17]. At the same time, Houttuynia cordata, white mustard seeds, etc. are used to relieve cough, reduce phlegm and relieve asthma, stir-fry chicken gold to strengthen the spleen and stomach, and improve appetite. Compatible with all prescriptions, strengthening the righteousness and eliminating pathogenic factors and applying both attack and supplementation, they have the effect of replenishing qi, nourishing essence, and strengthening the righteousness. They are used in combination to significantly improve symptoms and improve the quality of life.

In this study, the clinical symptom scores of the two groups after treatment were decreased compared with those before treatment, but the decrease was more obvious after treatment with Lung Cancer No. 1 prescription, which was significantly different from that of the control group after treatment. It can be seen that the treatment of lung cancer with traditional Chinese medicine can significantly improve clinical symptoms, improve the quality of life and tumor stability rate, and prolong the survival period. On the one hand, it can protect organs and reduce and prevent the damage of radiotherapy and chemotherapy to the body, and on the other hand, it can improve the body's immunity and increase the body's tolerance to radiotherapy and chemotherapy, thereby reducing tumor recurrence and metastasis [18].

Clinical studies have shown that new blood vessels provide a large amount of blood supply for the proliferation, invasion, and metastasis of tumor cells and play an important role in the occurrence and development of malignant tumors. VEGF can bind to vascular endothelial growth factor receptor 2 (VEGFR2) to mediate lymphatic and angiogenesis, participate in tumor angiogenesis and metastasis, and is closely related to the occurrence and development of SCLC tumors [19–22]. CYFRA21-1 is a soluble fragment of cytokeratin, which is widely distributed in lamellar or squamous epithelium. When tumor cells are lysed or necrotic, CYFRA21-1 can be released into the blood, which has a high diagnosis and efficacy evaluation for SCLC patients. CA125 is a polysaccharide protein with a very low concentration in the serum of healthy people. It is released into the blood when tumor infiltration occurs in the body. Its half-life is short and its metabolism is fast. Its detection level can be used to reflect the short-term efficacy of tumor treatment. CYFRA21-1 was all increased in patients with recurrent lung cancer, and the positive rate was 100%, indicating that its level changes can also be used as an auxiliary indicator for monitoring the recurrence of lung cancer. This clinical observation and study shows that the serum CYFRA21-1 content of the patients in the treatment group can be maintained at a low level. degree of progress [23–25]. The Lung Cancer No. 1 recipe can reduce the content of CYFRA21-1, and there is a significant difference compared with the control group. It can be seen that Lung Cancer No. 1 formula can improve the body's material metabolism and restore the yin-yang imbalance in the body by adjusting the level and expression of tumor markers. However, the level of tumor markers in the body decreased, the tumor burden was reduced, and various symptoms and signs of the corresponding patients were gradually relieved, indicating that reducing the tumor burden or inhibiting the activity of tumor cells may be one of the mechanisms of the curative effect of Lung Cancer No. 1 recipe [26].

The results of this study found that the levels of CYFRA21-1, CA125, and VGEF in the treatment group after treatment were significantly lower than those before treatment in the control group, indicating that PD-1/PD-L1 inhibitor chemotherapy combined with Lung Cancer Fang No. 1 therapy can effectively inhibit tumor cell proliferation and control of the condition of SCLC patients. This may be related to the fact that PD-1/PD-L1 inhibitor chemotherapy combined with Lung Cancer Fang No. 1 therapy can inhibit tumor cell proliferation and metastasis by inhibiting tumor angiogenesis [27–29]. The occurrence, development, and metastasis of tumors are closely related to the immune function of the body. The immune function of patients with malignant tumors is mostly in a suppressed state, and the body's antitumor ability and antitoxic side effects are weakened, which affects the prognosis of patients. Immune response is mediated by T lymphocytes. It is an important indicator for clinical evaluation of the immune function of the body [30–32]. CD3+ cells can enhance the body's antitumor immune response, and CD4+/CD8+ mainly reflects the killing activity of tumor cells. When malignant tumor occurs in the body, due to the secretion of certain factors, the content of CD3+, CD4+, and CD8+, especially the balance of CD4+/CD8+, is disturbed, leading to the disorder of immune response. It shows that Lung Cancer Fang No. 1 can reduce the incidence of adverse reactions in SCLC patients, improve the immune tolerance, and improve the immune function. Lung Cancer Fang No. 1 can enhance the body's antitumor effect and improve the patient's prognosis by reducing the body's immunosuppressive effect and enhancing the patient's resistance to adverse reactions [33]. The results of this study found that after treatment, the levels of CD3+ and CD4/CD8+ in the treatment group were significantly higher than those before treatment in the control group, and the total incidence of adverse reactions in the treatment group was significantly lower than that in the control group. All of these results suggest that Lung Cancer No. 1 mobilizes the patient's own antitumor ability, which may be due to the effect of tonic drugs such as Astragalus and American ginseng by enhancing the activity of peripheral blood NK cells and LAK cells and increasing the value of T3 and T4 lymphocytes [34, 35]. However, limitation included in the manuscript is that the mechanism of PD-1/PD-L1 inhibitor chemotherapy combined with Lung Cancer Fang No. 1 decreases the levels of CYFRA21-1, CA125, and VGEF which remains unknown, which will be investigated in further study.

## 5. Conclusion

In summary, to sum up, PD-1/PD-L1 inhibitor chemotherapy combined with Lung Cancer Fang No. 1 has a good and safe effect on SCLC patients, develops and improves the body's cellular immune function, adjusts the level and expression of tumor markers, improves the body's material metabolism, and restores the body's yin and yang imbalance.

## Figures and Tables

**Figure 1:** Clinical improvement. Before treatment, there was no significant difference in clinical improvement between the two groups. After treatment, the clinical symptom score (a) and weight change (b) of the treatment group were significantly improved. The clinical symptom score of the treatment group was lower than the control group and has higher body weight change. Values are mentioned as mean ± SD and analysed by employing one-way ANOVA followed by Tukey's multiple comparison post hoc test. The clinical symptom scores of the treatment group after treatment compared with before treatment was lower than the control group, but the weight change was higher than the control group (*P* < 0.05).

**Figure 2:** Comparison of tumor marker levels between the two groups of patients. Before treatment, there was no significant difference in tumor marker levels between the two groups. After treatment, CYFRA21-1 (a), CA125 (b), and VGEF (c) in the treatment group were significantly lower for the control group. Values are mentioned as mean ± SD and analysed by employing one-way ANOVA followed by Tukey's multiple comparison post hoc test. There were significant differences in tumor marker levels after treatment compared with before treatment (*P* < 0.05).

**Figure 3:** Comparison of immune levels in two groups of patients. The immune levels of the two groups of patients before treatment were comparable, while the CD4+ (a), CD3+ (b), and CD4+/CD8+ (c) after treatment were significantly different, and the treatment group was higher than the control group. Values are mentioned as mean ± SD and analysed by employing one-way ANOVA followed by Tukey's multiple comparison post hoc test. Compared with before treatment, the comparison of CD4+, CD3+, and CD4+/CD8+ in the treatment group was significantly different and higher than that before treatment in the control group (*P* < 0.05).

**Figure 4:** Comparison of clinical efficacy between the two groups of patients. After treatment, the clinical efficacy of the two groups was significantly improved. The DCR90.00% of the treatment group was significantly higher than that of the control group, 67.50%. The value was expressed as an integer, and chi-square comparison test was used. % was significantly higher than the control group (67.50% (*P* < 0.05)).

**Figure 5:** Comparison of prognostic complications between the two groups of patients. Analysis of complications after treatment showed that the fatigue, anorexia, hypertension, hand-foot syndrome, diarrhea, leukopenia, thrombocytopenia, and urinary protein of the patients in the treatment group were significantly lower than those in the control group, and the values were expressed as integers, and chi-square comparison test was used. Compared with before treatment, the treatment group was significantly lower than the control group (*P* < 0.05).

**Table 1:** Comparison of general data between the two groups $\left[n,\bar{x}\left(\pm s\right)\right]$.

Group	Gender (men/women)	Average age (age)	Tumor diameter (cm)	Pathological type		
				Squamous cell carcinoma	Adenocarcinoma	Squamous cell carcinoma
Control group (40)	28/12	36.63 ± 8.32	13.31 ± 1.67	10	22	8
Treatment group (40)	29/11	36.62 ± 8.31	13.33 ± 1.25	11	23	6
*χ* ^2^/*t*	0.061	0.007	0.074	0.065	0.051	0.346
*P*	0.805	0.995	0.941	0.799	0.822	0.556

## Data Availability

No data were used to support this study.

## References

[1] Owonikoko T. K., Dwivedi B., Chen Z. (2021). YAP1 expression in SCLC defines a distinct subtype with T-cell-inflamed phenotype. *Journal of Thoracic Oncology*.

[2] Lee S. S., Cheah Y. K. (2019). The interplay between microRNAs and cellular components of tumour microenvironment (TME) on non-small-cell lung cancer (NSCLC) progression. *Journal of Immunology Research*.

[3] Sager O., Dincoglan F., Demiral S. (2019). Utility of molecular imaging with 2-deoxy-2-[fluorine-18] fluoro-Dglucose positron emission tomography (18F-FDG PET) for small cell lung cancer (SCLC): a radiation oncology perspective. *Current Radiopharmaceuticals*.

[4] Lantuejoul S., Fernandez-Cuesta L., Damiola F., Girard N., McLeer A. (2020). New molecular classification of large cell neuroendocrine carcinoma and small cell lung carcinoma with potential therapeutic impacts. *Translational Lung Cancer Research*.

[5] García-González J., Ruiz-Bañobre J., Afonso-Afonso F. J. (2020). PD-(L)1 inhibitors in combination with chemotherapy as first-line treatment for non-small-cell lung cancer: a pairwise meta-analysis. *Journal of Clinical Medicine*.

[6] Liu C., Cui H., Gu D. (2017). Genetic polymorphisms and lung cancer risk: evidence from meta-analyses and genome-wide association studies. *Lung Cancer*.

[7] House C. M., Chinese Medical Association, Oncology Society of Chinese Medical Association (2018). Chinese Medical Association guidelines for clinical diagnosis and treatment of lung cancer (edition 2018). *Chinese Journal of Oncology*.

[8] Boran E., Ramantani G., Krayenbühl N. (2019). High-density ECoG improves the detection of high frequency oscillations that predict seizure outcome. *Clinical Neurophysiology*.

[9] Jonna S., Subramaniam D. S. (2019). Molecular diagnostics and targeted therapies in non-small cell lung cancer (NSCLC): an update. *Discovery Medicine*.

[10] Bennett B. M., Wells J. R., Panter C., Yuan Y., Penrod J. R. (2017). The humanistic burden of small cell lung cancer (SCLC): a systematic review of health-related quality of life (HRQoL) literature. *Frontiers in Pharmacology*.

[11] Li D., Xu X., Liu J. (2020). Small cell lung cancer (SCLC) incidence and trends vary by gender, geography, age, and subcategory based on population and hospital cancer registries in Hebei, China (2008–2017). *Thorac Cancer*.

[12] Wang S., Zimmermann S., Parikh K., Mansfield A. S., Adjei A. A. (2019). Current diagnosis and management of small-cell lung cancer. *Mayo Clinic Proceedings*.

[13] Kalemkerian G. P. (2016). Small cell lung cancer. *Seminars in Respiratory and Critical Care Medicine*.

[14] Chun S. G., Simone C. B., Amini A. (2021). American Radium Society appropriate use criteria: radiation therapy for limited-stage SCLC 2020. *Journal of Thoracic Oncology*.

[15] Ma W. P., Hu S. M., Xu Y. L. (2020). Haimufang decoction, a Chinese medicine formula for lung cancer, arrests cell cycle, stimulates apoptosis in NCI-H1975 cells, and induces M1 polarization in RAW 264.7 macrophage cells. *BMC Complementary Medicine and Therapies*.

[16] Kasymjanova G., Tran A. T., Cohen V. (2018). The use of a standardized Chinese herbal formula in patients with advanced lung cancer: a feasibility study. *Journal of Integrative Medicine*.

[17] Zheng T., Que Z., Jiao L. (2017). Herbal formula YYJD inhibits tumor growth by inducing cell cycle arrest and senescence in lung cancer. *Scientific Reports*.

[18] Spigel D. R., Socinski M. A. (2013). Rationale for chemotherapy, immunotherapy, and checkpoint blockade in SCLC: beyond traditional treatment approaches. *Journal of Thoracic Oncology*.

[19] Li H., Zhang Q., Wu Q. (2019). Interleukin-22 secreted by cancer-associated fibroblasts regulates the proliferation and metastasis of lung cancer cells via the PI3K-Akt-mTOR signaling pathway. *American Journal of Translational Research*.

[20] Meder L., Schuldt P., Thelen M. (2018). Combined VEGF and PD-L1 blockade displays synergistic treatment effects in an autochthonous mouse model of small cell lung cancer. *Cancer Research*.

[21] Hou C., Lu L., Liu Z., Lian Y., Xiao J. (2021). Resveratrol reduces drug resistance of SCLC cells by suppressing the inflammatory microenvironment and the STAT3/VEGF pathway. *FEBS Open Bio*.

[22] Zhao X., Sun X., Li X. L. (2012). Expression and clinical significance of STAT3, P-STAT3, and VEGF-C in small cell lung cancer. *Asian Pacific Journal of Cancer Prevention*.

[23] Xu Y., Fang W., Cheng B. (2020). Non-significant efficacy of icotinib plus pleurodesis in epidermal growth factor receptor positive mutant lung cancer patients after malignant pleural effusion drainage compared to icotinib alone. *Journal of Thoracic Disease*.

[24] Jiang Z. F., Wang M., Xu J. L. (2018). Thymidine kinase 1 combined with CEA, CYFRA21-1 and NSE improved its diagnostic value for lung cancer. *Life Sciences*.

[25] Liu L., Liu B., Zhu L. L., Li Y. (2013). CYFRA21-1 as a serum tumor marker for follow-up patients with squamous cell lung carcinoma and oropharynx squamous cell carcinoma. *Biomarkers in Medicine*.

[26] Han J., Hu J., Sun F., Bian H., Tang B., Fang X. (2021). Micro RNA-20a-5p suppresses tumor angiogenesis of non-small cell lung cancer through RRM2-mediated PI3K/Akt signaling pathway. *Molecular and Cellular Biochemistry*.

[27] Fields E. C., Rabinovitch R., Ryan N. E., Miften M., Westerly D. C. (2013). A detailed evaluation of TomoDirect 3DCRT planning for whole-breast radiation therapy. *Medical Dosimetry*.

[28] Longobardi B., De Martin E., Fiorino C. (2005). Comparing 3DCRT and inversely optimized IMRT planning for head and neck cancer: equivalence between step-and-shoot and sliding window techniques. *Radiotherapy and Oncology*.

[29] Dal Bello M. G., Filiberti R. A., Alama A. (2019). The role of CEA, CYFRA21-1 and NSE in monitoring tumor response to nivolumab in advanced non-small cell lung cancer (NSCLC) patients. *Journal of Translational Medicine*.

[30] Dochez V., Caillon H., Vaucel E., Dimet J., Winer N., Ducarme G. (2019). Biomarkers and algorithms for diagnosis of ovarian cancer: CA125, HE4, RMI and ROMA, a review. *Journal of Ovarian Research*.

[31] Pei Y., Changyuan G., Yuan L. (2018). Consistency of multi-platform detection of PD-L1 immunohistochemistry in biopsy specimens of advanced lung adenocarcinoma. *Chinese Journal of Pathology*.

[32] Xie J., Yang Q., He F. (2008). Effects of lung cancer no. 1 formula on immune function and serum VEGF and CYFRA21-1 in patients with advanced non-small cell lung cancer. *Chinese Traditional Chinese Medicine Journal of Information*.

[33] Zhu Z., Jianfeng S., Wei Z. (2019). Clinical observation of Fuzheng Yiai no. 1 formula combined with GP chemotherapy in the treatment of advanced non-small cell lung cancer based on the theory of “long illness and kidney”. *Chinese Medicine Pharmacology and Clinical*.

[34] Chen Q. J., Shi Y., Shi J. F. (2017). Liver X receptors agonist T0901317 downregulates matrix metalloproteinase-9 expression in non-small-cell lung cancer by repressing nuclear factor-*κ*B. *Anti-Cancer Drugs*.

[35] Shi H., Ji Y., Zhang D., Liu Y., Fang P. (2016). Micro RNA-3666-induced suppression of SIRT7 inhibits the growth of non-small cell lung cancer cells. *Oncol Rep.*.

